# Space Charge Dynamics in Epoxy Resins Under the Influence of a Long-Term High Electric Field at Various Temperatures

**DOI:** 10.3389/fchem.2022.904750

**Published:** 2022-06-15

**Authors:** Hongliang Zhang, Kun Li, Hai Jin, Kangle Li, Xiaonan Li, Peng Liu, Zongren Peng

**Affiliations:** ^1^ College of Electrical Engineering and Information Engineering, Lanzhou University of Technology, Lanzhou, China; ^2^ State Key Laboratory of Electrical Insulation and Power Equipment, Xi’an Jiaotong University, Xi’an, China

**Keywords:** space charge, epoxy resin, long term, temperature, bushing

## Abstract

As the main insulating material of an ultra-high voltage (UHV) resin impregnated paper (RIP) bushing, epoxy resin accumulates space charge under the DC voltage, which would affect the insulation properties of the bushing. In this article, the evolution of space charge accumulation and dissipation within the epoxy resin samples was measured under the influence of a long-term (24 h) electric field of 60 kV/mm at 40°, 60°, 80°, and 100°C. The experimental results show that the space charge transport in the epoxy sample was a long-time dynamic process. When the temperature was not greater than 60°C, only homocharge accumulation was observed within the samples, and the space charge distribution did not reach a stable state even after 24 h of voltage application. When the temperature was not lower than 80°C, the positive heterocharge accumulation was observed at the interface between cathode and epoxy. Through analysis by fitting and numerical simulation, it was verified that the positive heterocharge accumulation was caused by the limitation of the hole extraction, and the transport of holes within the samples obeyed the jump conductance model.

## Introduction

With ‘the one belt, one road strategy’ being proposed and pushed forward, the global energy Internet construction is in great potential demand. This is also an effective way to deal with the three major challenges, global resource shortage, environmental pollution, and climate change, and promote the sustainable development of a community with a shared future for mankind (Liu, 2016). China has a demand for interconnection with the neighboring national power grids, transcontinental transmission, and domestic long-distance transmission. The transmission distance required for a transnational and cross-regional interconnection may reach 5,000–6,000 km. The construction of the UHVDC transmission project will have great advantages in solving the long-distance transmission problem faced by the global energy Internet. Extrapolated according to the economic transmission distance, the voltage level of DC transmission should be between 1,500 and 1700 kV for such a long transmission distance (Liu, 2020). In order to prevent the threat of pollution and fire to the DC valve hall and meet the requirements of an oil-free valve hall, the valve side bushing of the UHV converter transformer in China adopts bushing with an epoxy resin impregnated paper (EIP) capacitor core (Chen et al., 2020). As the representative of the state-of-the-art technology, the EIP bushing poses many advantages such as high electrical strength, good heat resistance, strong partial discharge resistance, and good mechanical properties, which make it increasingly widely used in power systems. In addition, due to frequent oil leakage and gas production faults on the grid side of the converter transformer, which seriously endangers the converter and system operation safety, China is also promoting the replacement of 1,600–3150 A grid side bushing of the UHV converter transformer with an epoxy resin impregnated paper capacitor core (Xu et al., 2020).

In order to meet the severe operating conditions of UHV DC bushing, the epoxy formula system with a high glass transition temperature (126–140 °C) is required (Liu et al., 2015,^2016^). At high temperatures, high field, polarity reversal, and a rapid voltage change, the dielectric characteristics of epoxy composites show significant nonlinearity and the charge transport characteristics also vary significantly. This will lead to space charge accumulation and electric field distortion within EIP, which would accelerate the aging of insulating materials and may excite partial discharge, and even breakdown. Therefore, it is of great significance to study the space charge transport and accumulation characteristics of epoxy resin under extreme conditions for improving the levels of design, manufacture, operation, and maintenance of bushing. Liu et al. (2021) studied the effect of temperature and polarity reversal on space charge in epoxy composites and found that both the interface traps and space charge injection affect the space charge characteristics at different temperatures and field strengths. Wang et al. (2019)studied the problem of interface polarization in epoxy-impregnated paper insulation materials and proposed a method to evaluate the interface charge and electric field distribution under the action of different frequency voltages. Li et al. (2020) studied the space charge characteristics of epoxy materials at high temperatures and high field strengths and found that the ionization of an unreacted curing agent and electrode charge injection are the main sources of space charge. Awais et al. (2021) studied the epoxy composites suitable for high-frequency and high-temperature applications and found that the composite materials suitable for high-frequency and high-temperature environments can be obtained by controlling the stoichiometric ratio of epoxy and added nanofillers. Chillu et al. (2020) studied the space charge injection threshold and dissipation properties of aluminum–epoxy nanocomposites. Guvvala et al. (2020) studied the effect of thermal aging on the space charge characteristics of epoxy–aluminum nitride nanocomposites and successfully used laser-induced breakdown spectroscopy to distinguish the aging patterns. Haque et al. (2017) studied the charge detrapping and dipole polarization properties of epoxy by measuring the discharge current and identified the dipole polarization and space charge detrapping in the discharge current by using the Hamon approximation. Dong et al. (2017) found that nano-SiO_2_ can effectively inhibit the charge accumulation near the inner electrode of epoxy resin under isothermal or gradient conditions, which is mainly due to the enhancement of carrier extraction. Gao et al. (2016)found that the charge dissipation rate of LDPE/SiO_2_ nanocomposites was obviously slowed down, which was mainly due to the introduction of a large number of deep traps by nano-SiO_2_ (). Nelson and Fothergill (2004) studied the dielectric properties of the micro/nano-TiO_2_/epoxy composite system and they found that in the high-frequency range (>100 Hz), the dielectric constant of the microdoped composite system is the largest and the nanodoped composite system is the smallest (). There have been many studies on the space charge characteristics of epoxy materials under the action of short-term electric fields, but less research on the space charge characteristics of epoxy materials under the influence of long-term high electric fields.

With the rapid evolution in a short time, the space charge characteristics of epoxy composites under high temperatures and long-term high electric fields can better reflect their performance as the main insulation material of DC bushing in the long-term operation process. In this article, the space charge accumulation, migration, and dissipation characteristics of epoxy materials under high temperatures and long-term electric fields were measured by the pulsed electro-acoustic (PEA) space charge measurement system, and the influence of long-term electric field on the space charge transport process of epoxy materials was analyzed.

## Materials and Methods

### Preparation of Samples

In order to ensure the casting quality of the UHV DC bushing core, the epoxy material used should have good fluidity and wettability. In this article, bisphenol A diglycidyl ether (E51) was selected as the epoxy matrix, methylhexahydrophthalic anhydride (MeH-HPA) as the curing agent, and *N*,*N*-dimethylbenzylamine as the catalyst. after the E51 epoxy material, curing agent, and accelerator were mixed in a mass ratio of 100:85:0.3 and stirred at room temperature for about 20 min; then, the mixed solution was degassed in a 55°C vacuum oven for 6 h. Finally, the degassed mixed solution was poured into a steel mold under a vacuum to prepare for curing. The curing process adopts the step heating method. The solution was cured at 85°C for 4 h, and then at 110°C for 4 h, 145°C for 5 h, and 120°C for 4 h, and finally, cooled to room temperature naturally.

The size of the prepared sample was 110 mm × 110 mm × 0.24 mm. Using a differential scanning calorimeter DSC822e from METTLER TOLEDO, the glass transition temperature (*T*_g_) of the EP samples was measured to be about 140 °C with a temperature ramp of 10 K/min in the temperature range of 30°–200°C.

### Space Charge Measurement

The pulsed electro‐acoustic (PEA) space charge measurement system was composed of a programmable high-voltage power supply, nanosecond pulse power supply, RC pulse coupling circuit, test electrodes, piezoelectric sensor, signal acquisition, and processing system. The programmable high-voltage power supply consists of TTi TGA1241 programmable signal generator and Trek 30 kV/20 mA high-voltage power amplifier. The latter has a self-protection function, which can automatically cut off the high-voltage output to ensure the safety of the experimental system when the sample was broken down. The half-peak pulse width of the nanosecond pulse power supply is about 5 ns and the repetition rate is 153.8 Hz. A polyvinylidene fluoride trifluoroethylene (P (VDF TrFE)) film with a thickness of 12 μm was used as the piezoelectric sensor, in which the curie point temperature is about 135°C.

In order to ensure good contact between the sample and the test electrode and eliminate the influence of electrode material on the space charge dynamics, gold electrodes with a diameter of 16 mm are sputtered on both sides of all the tested epoxy samples. The samples with sputtered gold electrodes were dried in a 105°C vacuum oven for 12 h before testing to fully eliminate the influence of moisture. The sample was immersed in silicone oil during measurements to enhance the acoustic coupling between the sample and the electrode and eliminate partial discharge under a high electric field. The migration rate of the space charge inside the EP samples was accelerated at a high temperature and the dynamic change of the space charge was evident. In order to improve the efficiency of the experiment, an electric field of 60 kV/mm was continuously applied to the epoxy samples for 24 h (1,440 min) at temperatures of 40°, 60°, 80°, and 100°. The dynamics of space charge during polarization and depolarization were measured by the PEA space charge measurement system.

### Bipolar Carrier Transport Model

A bipolar charge transport model has been widely used to study the relationship among charge transport, accumulation characteristics, polymer conductivity, surface potential attenuation, breakdown, and other processes (Chen and Wang, 2013). In dielectrics, the dynamic behavior of charges mainly includes processes such as injection, trapping, detrapping, and recombination. Figure 1 shows a schematic diagram of a one-dimensional simulation model of the bipolar charge transport. The physical process is as follows: when a DC voltage is applied, the carriers are injected from two electrodes. Holes and electrons migrate in the opposite direction, which is relative to the electric field inside the sample. In the process of migration, some electrons/holes migrate in the conduction/valence band through hopping conductance, and some electrons/holes are trapped by deep traps. The free charge (free hole/free electron) and trapped charge (trapped electron/trapped hole) with different polarities will recombine and release energy. The difficulty in recombination depends on the energy level difference between them. Some carriers migrating at the interface between the sample and electrode can be successfully extracted, while others are blocked and accumulated due to the existence of an interface barrier. The thickness of the sample is *d*, where x = 0 is grounded and x = d is connected to the high-voltage electrode. In order to simplify the analysis, the simulation conditions are set as the applied field strength of 60 kV/mm for 2 h at temperatures of 40°, 60°, 80°, and 100°C.

**FIGURE 1:** Schematic diagram of bipolar charge transport mode.

Charge injection at anode and cathode follows Schottky’s law, and its expression is

$$\begin{array}{c} j_{\mathrm{hi}/\mathrm{ei}}\left(x,t\right)=AT{\left(x\right)}^{2}\exp\left(\frac{-e\omega_{\mathrm{ei}/\mathrm{hi}}}{kT\left(x\right)}\right)\exp\left(\frac{e}{kT\left(x\right)}\sqrt{\frac{e\left|E\left(x,t\right)\right|}{4\pi \varepsilon_{0}\varepsilon_{r}}}\right) \end{array},$$ (1)

where *j*_hi_ and *j*_ei_ are the injection current densities of the cathode (x = 0) and anode (x = d), respectively, *T(0)* and *T(d)* are the temperatures of the cathode and anode, respectively, *w*_ei_ and *w*_hi_ are the injection barriers of the electron and hole at the interface, respectively, *k* is the Boltzmann constant, and *A* is the Richardson constant.

The carrier extraction limitation is also defined in the Schottky form as follows:

$$\begin{array}{c} j_{\mathrm{ho}/\mathrm{eo}}\left(x,t\right)=AT{\left(x\right)}^{2}\exp\left(\frac{-e\omega_{\mathrm{eo}/\mathrm{ho}}}{kT\left(x\right)}\right)\exp\left(\frac{e}{kT\left(x\right)}\sqrt{\frac{e\left|E\left(x,t\right)\right|}{4\pi \varepsilon_{0}\varepsilon_{r}}}\right) \end{array},$$ (2)

where *j*_ho_ and *j*_eo,_ respectively, represent the extraction current density of the cathode/anode, *w*_ho_ and *w*_eo,_ respectively, represent the extraction barriers of electron and hole at the interface.

The carrier migration is determined by the current continuity equation, the charge transport equation, and the Poisson equation, which are expressed as follows:

$$\begin{array}{c} \{\begin{array}{c} \frac{\partial n\left(x,t\right)}{\partial t}+\frac{\partial j\left(x,t\right)}{\partial x}=s_{a}\left(x,t\right)\\ j\left(x,t\right)=\mu \left(x,t\right)n\left(x,t\right)E\left(x,t\right)\\ \frac{\partial E\left(x,t\right)}{\partial x}=\frac{\rho \left(x,t\right)}{\varepsilon }, \end{array} \end{array}$$ (3)

where *ρ* is the net charge density and *S*_*i*_ is the source term that represents the interaction between the carriers. The space charge distribution in the sample can be obtained by solving the above three equations simultaneously.

## Results

### Space Charge Profiles Under the influence of Long-Term High Electric Field Strength at Various Temperatures

The space charge profiles within the epoxy samples under the influence of a long-term electric field of 60 kV/mm at various temperatures are shown in Figure 2. It can be seen from the figure that the space charge profiles at 40° and 60°C are similar. In the first 1 h of voltage application, the injection of space charge was not obvious at 40° and 60°C. Afterward, the position of the space charge peak near the lower electrode moved slightly toward the inside of the sample, and the magnitude of the charge peak decreased slightly during the movement as the time of voltage application increased. This indicates that s injection of charges appeared within the samples.

**FIGURE 2:** Space charge profiles at different times at 60 kV/mm and various temperatures.

When the temperature was higher than 80°C, the negative homocharge injection near the lower electrode obviously appeared within the sample in the first hour of applying the voltage. Due to the smaller injection barrier of the electron than that of the hole, more electrons were injected into the sample at a high temperature. The negative homocharge near the cathode had disappeared to some extent after the third hour of voltage application at 100°C, which was observed at 80 °C after the 12th hour. This shows that with the increase of voltage application time and temperature, the migration speed of the hole in the sample was gradually accelerated and some electrons near the lower negative electrode were neutralized by recombination with the holes. Accompanied by the disappearance of the negative homocharge, an accumulation of positive heterocharge occurred near the lower electrode. After 24 h of voltage application, the positive heterocharge near the lower electrode continued to increase, which indued more surface charges on the lower electrode. On the whole, when the temperature was not greater than 60°C, the curve distribution was relatively flat, which indicates that the carrier transport processes such as trapping and detrapping were not obvious and the migration speed was relatively slow. When the temperature was greater than or equal to 80°C, the peak value at the two electrodes became larger, which indicated that a high temperature promotes the process of carrier injection and migration.

The space charge profiles at various temperatures in the process of removing voltage are shown in Figure 3. It can be seen from the figure that the space charge profiles at various temperatures show a great difference. When the temperature was 40°C, there were only negative homocharges that appeared near the lower electrode and no positive homocharges were observed near the upper electrode.

**FIGURE 3:** Space charge profiles at different times after removing voltage at various temperatures.

More negative homocharges were injected at 60°C than at 40°C. Positive homocharges were also observed near the upper electrode where the amount was smaller than that of negative homocharges near the lower electrode. The injected space charge peak and the induced charge peak on the electrode were distributed on both sides of the electrode when the temperature was not greater than 60°C.

At a temperature of 80°C, the peak value of negative homocharges near the lower electrode was evidently smaller than that at 60°C, in which the distribution width within the sample was very wide. Since the PEA space charge measurement can only measure the net charge, it is impossible to measure whether the charge exists or not when the distance between the different polarity charges is shorter than the spatial resolution of the measuring device. However, if the induced charge peak of the lower electrode appeared in the samples, it can still be inferred that this was caused by the overlap of the positive induced charge profile on the lower electrode and the positive heterocharge profile near the lower electrode. At the same time, the positive heterocharge near the lower electrode may offset the amount of negative charge injected by the lower electrode, which leads to a decrease in the negative charge peak.

At 100°C, the positive space charge was only observed within the sample. The peak of the positive charge profile near the lower electrode was slightly higher than that near the upper electrode after 1 min of removing the voltage. After 1h, the peak of the positive charge near the upper electrode decreased significantly, while the peak near the lower electrode did not vary significantly.

Comparing Figure 3A with Figure 3B, it can be seen that each peak value of space charge distribution within the epoxy sample only slightly decreased after 1 h of removing the voltage, except at 100°C. This indicates that it would take a longer time for the space charge to dissipate. The profiles of space charge in the thickness of less than 0 μm represent the induced charge at the electrode by the internal space charge of the samples. At temperatures not greater than 60°C, the induced charge was positive due to the negative homocharges accumulated in the samples. When the temperature was 80°C, the positive heterocharges began to accumulate near the lower electrode, where the amount was still less than that of the negative homocharges. Thus, the profile of the induced positive charge at the lower electrode merged with that of the positive heterocharge, which shifts the positive charge peak into the sample. When the temperature was 100°C, the amount of residual positive charges exceeded that of the negative charges, which induced negative charges at the lower electrode and the negative charge profile had a thickness less than 0 μm.

### Electric Field Distortion in Epoxy Samples at Various Temperatures

The distortion degree of the electric field within the epoxy samples can be calculated as follows:

$$\begin{array}{c} F_{d}=\frac{\left|E_{\text{max}}\right|-\left|E_{a}\right|}{\left|E_{a}\right|}\times 100\% \end{array},$$ (4)

where *E*_max_ is the maximum field strength in the sample and *E*_a_ is the average field strength of the applied voltage.

The electric field distortions within the epoxy samples at various temperatures were calculated by the previous formula, which is shown in Figure 4A. At the same time, the change in the position of the maximum field intensity in the sample with time is made, as shown in Figure 4B.

**FIGURE 4:** Distortion of the internal electric field with time at 60 kV/mm and various temperatures. **(A)** Electric field distortion, **(B)** Variation of the position of the maximum electric field.

It can be seen from Figure4A that the electric field distortion was small at 40 °C and it increased slightly with time and the maximum electric field distortion was about 14.74%. Within the first 100 min of voltage application, the maximum field strength was scattered in the middle and lower parts of the sample, then quickly appeared near the lower electrode, and slightly moved into the sample with time.

When the temperature was 60°C, the electric field distortion increased obviously with time, and the maximum distortion rate was about 40.87%. Within 200 min of voltage application, the position of the maximum field intensity gradually moved from the middle and lower parts to the middle and upper parts within the sample with time, which finally appeared at a position slightly above the middle part of the sample.

When the temperature was 80°C, the electric field distortion first increased rapidly with time and then decreased slightly after about 600 min. The maximum distortion rate was about 49.11%. The position of the maximum field strength appeared stable near the upper electrode.

When the temperature was 100°C, the distortion rate of the electric field in the sample varied slowly and the maximum field strength appeared near the upper electrode within the first 300 min. The distortion rate of the electric field at 100°C was slightly smaller in the first 600 min than that at 80°C. After applying voltage for about 300°min, the distortion rate of the electric field increased obviously with the increase of time, and its maximum value was about 54.01%, and the maximum electric field shifted accordingly from the area near the upper electrode to the area near the lower electrode.

## Discussion

### Space Charge Transport Mechanism of Epoxy Materials at Various Temperatures

Epoxy resin is a kind of macromolecule polymer, in which amorphous and crystalline forms coexist. With the deepening research on the phenomenon of space charge in polymer, it is now considered that injection and extraction of negative charge (electron) and positive charge (hole) occur simultaneously at the interface between the electrode and polymer. Accordingly, the charge transport within the polymer is also accomplished by the migration of electrons and holes. The migration process of electrons and holes in a polymer can be described by the bipolar carrier transport model (Min and Li, 2014; Li, 2015).

On the whole, the atomic distribution of the polymer is irregular but it is regular in local areas. The energy band formed by the periodic arrangement of atoms can only exist in each local region, which is interrupted in the irregular atomic distribution region. Traps will be formed in regions with discontinuities in the band, with the trapping electrons and holes. The traps can be divided into deep traps and shallow traps according to the energy required for carrier detrapping. The time of carrier trapping and detrapping in the shallow trap is much shorter than the response time of the PEA space charge measuring device, so the time of carrier trapping and detrapping in the shallow trap can be ignored (Liu and Chen, 2013; Li et al., 2016). The carriers stay in the deep traps for a long time, so the space charge measured by the PEA device can be considered as the carriers trapped by the deep trap.

By analyzing the space charge characteristics and electric field distribution of epoxy materials at various temperatures under the influence of a long-term electric field of 60 kV/mm, it can be seen that the temperature had an obvious influence on the space charge injection and migration in epoxy materials. Therefore, the charge transport process at the electrode/epoxy interface should mainly obey the thermionic emission process enhanced by the electric field. When the temperature was not greater than 60°C, the negative charge (electron) was mainly injected into the epoxy sample, and the injected positive charge is relatively less. This indicates that the interface barrier of the epoxy/electrode interface for electron injection was lower than that for hole injection at lower temperatures (not greater than 60°C). When the temperature was not lower than 80°C, the electron and hole injection in the samples became obvious, which indicates that with the increase in temperature, the carrier in the electrode gain higher energy and can be injected into the sample more easily.

When the temperature was not lower than 80°C, with increasing time of the applying voltage, the positive charges accumulate near the cathode within the sample. With the increase in temperature, the amount of accumulated positive charges exceeds that of the negative charges in the sample. Only positive heterocharges were observed after a long time at high fields and high temperatures and it can be inferred that limiting of hole extraction occurred at the interface between the epoxy and cathode.

The accumulation of positive heterocharges can be analyzed by hopping conductance theory. Assuming that the migration rate of the hole in the direction of the electric field is *v*_d_ (Dissado and Fothergill, 1992),

$$\begin{array}{c} v_{d}=a\upsilon e^{-\frac{\Delta }{k_{B}T}}\times 2\sinh\left(\frac{Eaq_{e}}{2kT}\right) \end{array},$$ (5)

where *a* is the average single hopping distance of the hole; υ is the thermal vibration frequency of the hole; *Δ* is the trap depth; *k* = 1.38 × 10–23 J/K is the Boltzmann constant; *T* is the absolute temperature; *E* is the applied electric field intensity; and *q*_*e*_ is the charge quantity. In this article, it is considered that each charge is univalent, that is, *q*_*e*_ = 1.6 × 10–19 C.

In this article, the following formula is used to estimate υ (Tzimas et al., 2010):

$$\begin{array}{c} \upsilon =\frac{kT}{h} \end{array},$$ (6)

where *h* = 6.63 × 10–34 Js is the Planck constant. Because *υ* does not change much with temperature, the corresponding value at 100°C is taken in the analysis, that is, *υ* = 7.76×10^12^.

According to the results of the space charge test in Figures 2, the time when the distinguishable positive charge just appeared in the area near the lower electrode in the sample was taken as the time when the holes migrated through the whole sample. In this way, after the hole migration rate *v*_d_ is determined from the sample thickness and migration time, the relevant parameters of the hole hopping migration process can be obtained by the fitting analysis with formulae (2–18), as shown in Table 1.

**TABLE 1:** Related parameters of hole hopping migration in the epoxy samples at 60 kV/mm.

Temperature/°C	Migration Time/min	*v*_d_/(μm/s)	Δ/eV	*a*/Nm
80	753	0.0053	1.29	12.25
100	118	0.034	1.29	12.25

Substituting the fitting results from Table 1 into Eq. 5, we get the fitting curve of the hole migration rate with temperature in the epoxy sample, as shown in Figure 5.

**FIGURE 5:** Variation of migration rate of holes in the epoxy samples with temperature.

From the fitting results, it can be seen that the hopping conductance model fits the hole mobility measured by space charge well with the change of temperature. At the same time, it shows that the change between them accords with the Arrhenius relation. Due to the three-dimensional network structure and complex microstructure of the epoxy material after curing, the specific migration path of the electrons and holes in the epoxy material cannot be clearly explained at present. From Eq. 5, it can be seen that the migration of holes in the epoxy material is not only affected by the temperature but also affected by the electric field intensity, so it is necessary to further analyze the influence of the electric field change on the space charge characteristics in the epoxy materials. In addition, by analyzing the dissipation characteristics of the space charge in epoxy samples, the trap-related parameters in the sample can be obtained in more detail. However, from the previous measurement results, it can be seen that the residual space charge in the epoxy sample after depressurization is difficult to dissipate in a short time, so it is necessary to extend the measurement time of the space charge distribution after removing the applied voltage to obtain more detailed space charge characteristic data.

### Numerical Simulation of Space Charge

Combined with the measurement results of the space charge experiment, the parameters of the epoxy simulation model are determined, as shown in Table 2.

**TABLE 2:** Parameter values of the bipolar carrier transport model.

Parameter	Value	Unit
$B_{e}/B_{h}$ (Detrapping coefficient)	0.025	$s^{-1}$
$S_{e\mu ,ht}/S_{et,h\mu }/S_{et,ht}$ (Different polarity carrier recombination coefficients)	$1\times 10^{-5}$	$m^{3}\cdot {\left(s\cdot C\right)}^{-1}$
$w_{ei}$	1.17	eV
${\text{w}}_{hi}$	1.2	eV
${\text{w}}_{eo}$	1.2	eV
${\text{w}}_{ho}$	1.5	eV
$N_{eot}/N_{hot}$ (Trap density)	100	$C\cdot m^{-3}$
$\mu_{e}/\mu_{h}$	4 × 10–15/2 × 10–15	$m^{2}\cdot {\left(v\cdot s\right)}^{-1}$

Figure 6 shows the dynamic revolutions of the space charge profiles at different times at various temperatures. It can be seen from the figure that the space charge distribution at 40°–60°C is roughly similar, showing the same homocharge distribution. At 40°C, the space charge injection near the two electrodes is not obvious in the first 100 s of the applied voltage. With the extension of the applied voltage time, the injection of space charge increases gradually and the diffusion range of negative charges is larger than that of positive charges. At 60°C, with the increase in temperature, the charge accumulation of the two electrodes increases rapidly in the first 100 s, which indicates that the increase in temperature strengthens the injection of carriers and traps a large amount of charges t near the electrodes.

**FIGURE 6:** Distribution of space charge in the epoxy samples at60 kV/mm for different times at various temperatures.

When the temperature is 80°C, it can be clearly seen that the heterocharge accumulation began to appear at 0–15 μm near the cathode around 3000 s, which gradually decreased with the thickness direction and then turned into the homocharge accumulation. This shows that the positive charge transported to the vicinity of the cathode cannot be extracted due to interface blocking. At this time, the positive charge accumulation of the cathode is greater than the negative charge accumulation, which makes the positive charge diffuse into the sample; and at the same time, a large amount of injected electrons cover up the positive charge again.

When the temperature is 100°C, the time when the heterocharge begins to accumulate is further advanced. It shows that with the increase of temperature, the migration rate and injection amount of holes also increase. In addition, it can be seen that from 40 to 100 °C, the anode has never accumulated negative charges, indicating that the holes are easier to be extracted than electrons.

From the distribution of space charge, the electric field distribution can be obtained from the following formula, and the result is shown in Figure 7 as follows:

$$\begin{array}{c} E\left(x\right)=\frac{1}{\varepsilon_{0}\varepsilon_{r}}\int_{x_{0}}^{x}\rho \left(x\right)dx \end{array}.$$ (7)

**FIGURE 7:** Electric field distribution in the epoxy samples at 60 kV/mm for different times at various temperatures.

It can be seen from Figure 7 that the electric field distribution at 40–60 °C is similar. The electric field distortion is not obvious within 100 s of the initial applied voltage. With the extension of the applied voltage, the degree of electric field distortion gradually increases, and the degree of distortion near the two electrodes is greater than that in the middle of the sample. The maximum field strengths at 40° and 60°C are 66 and 71 kV/mm, respectively.

When the temperature is 80°C, it can be seen that the degree of electric field distortion in the sample is further increased. The maximum field strength tends to migrate toward the middle of the sample near the cathode. This shows that the migration depth of negative charges injected by the cathode is greater than that of positive charges. When the temperature reaches 100°C, the degree of electric field distortion in the sample increases significantly. When the applied voltage reaches 2000 s, the maximum field strength is as high as 112 kV/mm. This shows that the charge injection amount and migration rate of the two electrodes increase to different degrees at high temperatures, which eventually leads to the dynamic change of space charge distribution, thus greatly affecting the electric field distribution.

Based on the abovementioned numerical simulation results of charge distribution and electric field distribution, it can be seen that at different temperatures, the distribution trend of space charge obtained by the experiment and simulation is basically consistent. When the temperature is less than or equal to 60°C, the space charge distribution is the homocharge accumulation, and the degree of electric field distortion is small. When the temperature is greater than or equal to 80°C, the accumulation of heterocharge begins to appear. The time of accumulation of heterocharge at 100°C is less than that at 80°C and the degree of electric field distortion at this time is evidently increased.

## Conclusion

In this article, epoxy resin samples were prepared according to the epoxy composite formulation used in UHVDC voltage bushing. The space charge profiles and internal electric field distribution in epoxy samples under the influence of a long-term (24 h) electric field of 60 kV/mm at various temperatures were measured. After analyzing and simulating the dynamics of space charge accumulation, migration, and dissipation, some conclusions are summarized as follows:

1) When the temperature was not greater than 60°C, only homocharge accumulation was observed in the epoxy samples at 60 kV/mm, and the amount of injected electrons was significantly larger than that of the injected holes. In addition, the process of space charge accumulation did not reach a stable distribution within 24 h.
2) When the temperature was not lower than 80°C, positive heterocharges were observed within the samples near the cathode at 60 kV/mm. The relationship between the time of appearance of positive heterocharges and temperatures obeyed the hopping conductance model, in which the depth was around 1.29 eV and the hopping distance was around 12.25 nm.
3) The numerical simulation results were consistent with the experimental results, which proved that the limitation of hole extraction existed at the interface between the epoxy and cathode at high temperatures and high electric fields.

## Data Availability

The raw data supporting the conclusion of this article will be made available by the authors, without undue reservation.
